RETRACTED

# Long Noncoding RNA SNHG12 Promotes Prostate Tumor Occurrence and Progression via AKT Regulation

**DOI:** 10.1155/2020/8812923

**Published:** 2020-12-22

**Authors:** Zheng Chen, Tao Qi, Xiao-ping Qin, Jue Wang, Zhang-sen Huang, Xiao-yong Hu, Guo Chen, Li-jun Qu, Yu-min Zhuo

**Affiliations:** ^1^Department of Urology, The First Affiliated Hospital of Jinan University, Guangzhou 510632, China; ^2^Department of Infertility and Sexual Medicine, The Third Affiliated Hospital of Jinan University, Guangzhou 510630, China; ^3^Department of Pathology, The First Affiliated Hospital of Sun Yat-sen University, Guangzhou 510080, China; ^4^Department of Urology, The Sixth People's Hospital Affiliated of Shanghai Jiaotong University, Shanghai 200000, China

## Abstract

The small nucleolar RNA host gene 12 (SNHG12) has been reported to play an important role in the tumorigenesis and progression of PCa, but the functional underlying mechanism has not been studied clearly. We detected the expression level of SNHG12 in PCa tissues and matched adjacent normal tissues that were collected from 85 patients. Then, colony formation assays, MTT experiments, and flow cytometry were used to examine the effect of SNHG12 on proliferation, cell cycle distribution, and apoptosis of DU145 cells. Further, Transwell invasion assay was utilized to assess whether SNHG12 participates in PCa cell invasion and affects the secretion of VEGF secretion in DU145 cells. Finally, we investigated the effect of SNHG12 on tumor growth *in vivo*. We found that SNHG12 promoted cell proliferation and suppressed apoptosis in PCa cells, which suggests that SNHG12 is probably a novel PCa biomarker and therapy target of PCa.

## 1. Background

Prostate cancer (PCa) is the second most frequent diagnosis male malignancies and the leading cause of death worldwide [1, 2]. In China, PCa is one of the top ten leading causes of cancer-related death among men, and the morbidity and mortality rates of PCa are increasing annually rapidly, which is a serious risk to men's life [3–6]. Even with the medical condition improving, the 5-year survival rate of PCa patients is still low [3, 6]. Therefore, further studying the mechanism underlying the pathogenesis and progression of PCa is very important and necessary.

Previous epidemiology of PCa studies have shown that the pathogenesis of PCa is closely associated with age, heredity, diet, environment, sex hormones, and epigenetic changes [7, 8]. Changes in epigenetics have been increasingly recognized as important factors in the occurrence and development of PCa [9, 10]. The most common epigenetic changes include the dysregulation of long noncoding RNAs (lncRNAs) [11], which are transcribed by RNA polymerase II and have more than 200 nucleotides without protein-coding ability [12]. For instance, the lncRNA CCAT1 promoted PCa cell proliferation by interacting with DDX5 and miR-28-5p [13]. Knockdown of lncRNA SNHG7 inhibited epithelial-mesenchymal transition in PCa through the miR-324-3p/WNT2B axis *in vitro* [14]. High lncRNA FEZF1-AS1 expression promoted cell proliferation and metastasis through Notch signaling in PCa [15]. Therefore, understanding the effects of lncRNAs on PCa could help identify novel diagnostic and therapeutic targets [16, 17].

RETRACTED

Recently, lncRNAs have been found to be closely associated with tumorigenesis, growth, progression, and metastasis, as they act as gene regulators via transcriptional pathways [18]. For instance, lncRNA host gene 12 (SNHG12) is considered a potential therapeutic target and biomarker of various human cancers, which is upregulated in gastric cancer, non-small cell lung cancer, triple negative breast cancer, and so on [19–21]. Recently, SNHG12 was reported to promote cell proliferation and accelerate tumorigenesis of PCa [22, 23]. However, effects of SNHG12 on the tumorigenesis and progression of PCa have not been studied clearly, and the mechanism underlying SNHG12 promote PCa cell proliferation needs to be further investigated.

Our study investigated whether SNHG12 exerts strong oncogenic effects during the progression of PCa cells. To this end, we explored (i) the effects of SNHG12 on PCa cell proliferation, cell cycle progression, and apoptosis; (ii) the underlying mechanism; and (iii) the impact of SNHG12 on angiogenic tube formation and vascular endothelial growth factor (VEGF) secretion in a human PCa cell line (i.e., DU145). Our results suggested that SNHG12 could be a novel molecular biomarker for PCa and provide a possible clinical therapeutic strategy for PCa.

## 2. Materials and Methods

### 2.1. Patients and Tissue Samples

Eighty-five pairs of PCa samples and control samples (i.e., matched normal prostate tissues) were derived from patients (*N* = 85) of primary PCa who underwent surgery at the Department of Urology of the First Affiliated Hospital of Jinan University and the Sixth People's Hospital Affiliated with Shanghai Jiao Tong University. The samples were washed with sufficient cold phosphate-buffered saline (PBS) to reduce blood contamination and were then immediately placed in liquid nitrogen until for further experiments.

The patient was selected if he/she (i) was preoperatively diagnosed as low-risk PCa according to NCCN guidelines (PSA ≤ 10 ng/ml, GS score ≤ 6, T ≤ T2a) [18] and thus not diagnosed as adenocarcinoma of PCa or specific pathological types of PCa (e.g., ductal cancer, lymphoma, endocrine cancer of the prostate, and sarcoma), (ii) had punctured at least 8 stitches during the surgery when samples were taken, (iii) had not received endocrine therapy, radiotherapy, or chemotherapy, (iv) had no surgical contraindications or other types of tumors and not received radical PCa surgeries before this operation, and (v) had complete records of preoperative case data. All the above criteria should be met for each selected patient.

RETRACTED

The protocol was approved by the Ethic Committee (Clinical Management Committee) of the First Affiliated Hospital of Jinan University, the Sixth People's Hospital Affiliated with Shanghai Jiao Tong University and complied with world Medical Association Declaration of Helsinki. Written informed consents were obtained from all patients.

### 2.2. Cell Culture

The human prostate matrix immortalized WPMY-1 cells and human prostate cancer cell lines LNCAP, DU145, and PC-3 were purchased from the American Type Culture Collection (ATCC) and were cultured in Dulbecco's Modified Eagle's Medium (DMEM) supplemented with 10% fetal bovine serum (FBS) (Invitrogen, Carlsbad, CA) and 2 mmol/l L-glutamine, 100 U/ml penicillin, and 100 *μ*g/ml streptomycin. All cell lines were maintained under standard cell culture conditions at 37°C in an incubator with 5% CO_2_ and 95% air and were passaged with 0.25% trypsin (Sigma, USA) for digestion and subculture when the cells were approximately 90% confluent. Additionally, the certificate of cell authentication is provided in the supplementary material.

### 2.3. Lentiviral shRNA-Mediated Knockdown

Lentiviral shRNA plasmids with microRNA scaffolds (Neuron Biotech, Shanghai, China) targeting human SNHG12 (hereafter referred to as lenti-EGFP-SNHG12-miR plasmids) or containing scrambled shRNA (hereafter referred to as lenti-EGFP plasmids) were constructed. Cells (at a density of 1.0 × 105/ml) were cultured in 2 ml medium without antibiotics in 6-well plates. When the cells were ~80% confluent, the above-mentioned plasmids were transfected into cells using Lipofectamine 2000 (Invitrogen) together with gag/pol packaging vectors and VSVG-encoding plasmids to produce lentiviruses according to the manufacturer's recommendations. Moreover, the multiplicity of infection (MOI) of lentivirus-plasmids in target cells was 10. A volume of 5 *μ*l of Lipofectamine 2000 was diluted with 250 *μ*l of serum-free medium (Opti-MEM, Gibco, Invitrogen, USA), incubated for 5 min at room temperature, and swirled gently to mix evenly, after which the plasmids described above were added; this mixture was then incubated for 20 min at room temperature. The mixture was eventually added to the cell culture plates, which were incubated at a temperature of 37°C in a humidified incubator with 95% O_2_ and 5% CO_2_. After an additional 6~8 h incubation, the mixture was replaced by complete medium, and the cells were incubated for 24~48 h.

RETRACTED

### 2.4. Quantitative Reverse Transcription-Polymerase Chain Reaction (qRT-PCR) Detection

The total RNA of tumor tissue samples and cultured cells was extracted using TRIzol reagent (TIANGEN, China) in accordance with the manufacturer's instructions. The RNA preparations were then cleared of genomic DNA contaminants by DNase treatment (Thermo, USA). Then, the concentration and purity of the RNA samples were assessed by spectrophotometrically determining the optical density ratio, and single-strand complementary DNA (cDNA) was synthesized from 0.5 *μ*g of total RNA using a PrimeScript RT reagent kit (Takara, Japan) according to a standard protocol. Quantitative analysis of SNHG12 was performed on a 7500 Fast Real-time PCR system (Applied Biosystems, USA) using a SYBR® Premix Ex Taq™ II (TliRNaseH Plus) kit according to the manufacturer's manual with 0.1 *μ*g cDNA. The PCR temperature conditions were as follows: 1 cycle of denaturing at 95°C for 30 s, 40 cycles of denaturing at 95°C for 5 s, annealing at 60°C for 34 s (with data collection at the end of the 60°C step at each cycle), and dissociation at 95°C for 15 s, 60°C for 1 min, and 95°C for 15 s. Glyceraldehyde 3-phosphate dehydrogenase (GAPDH) was used as an internal control to normalize the SNHG12 quantitative data, which were further calculated with the 2^−*ΔΔ*Ct^ method. The sequences of the primers used for qRT-PCR were as follows: SNHG12, 5'-TCTGGTGATCGAGGACTTCC-3' (forward) and 5'-ACCTCCTCAGTATCACACACT-3' (reverse); GAPDH, 5'-ACACCCACTCCTCCACCTTT-3' (forward) and 5'-TTACTCCTTGGAGGCCATGT-3' (reverse).

### 2.5. Western Blot Analysis

After collection, the cells were lysed in lysis buffer (Beyotime, Shanghai, China) supplemented with a “cocktail” of phenylmethylsulfonyl fluoride, phosphatase inhibitor, and protease inhibitor. The protein concentration of each sample was measured using the BCA protein assay kit (Pierce Biotechnology, USA) following the manufacturer's guidelines. Then, equivalent quantities of protein (30 *μ*g) were separated on 8~15% discontinuous SDS-polyacrylamide gels for electrophoresis (SDS-PAGE) and transferred onto nitrocellulose (NC) blotting membranes. The membranes were blocked with 10% skim milk for 2 h at room temperature and incubated overnight at 4°C with the appropriate primary antibodies. The membranes were then washed and further incubated with secondary antibodies (horseradish peroxidase conjugated) at room temperature for 1 h. The secondary antibodies were visualized with an enhanced chemiluminescence (ECL) system (Pierce Biotechnology, Rockford, IL). The band grayscale and the ratio of the band intensity of each protein of interest to those of the loading control were detected with the Adobe Photoshop software.

RETRACTED

### 2.6. Colony Formation Assay

Cell monolayers were dissociated into single cells, which were then seeded into 6-well plates at a density of 500 cells/well in triplicate wells 4 days after transfection. After the fourteenth passage, the cells were fixed in methanol and stained with 0.5% crystal violet. The colony formation rate was calculated by dividing the number of colonies by the number of seeded cells.

### 2.7. Flow Cytometry Assay

For flow cytometry, cells in the logarithmic growth phase were harvested by trypsinization one week after lentivirus infection, fixed in 70% (*v*/*v*) ethanol overnight at -20°C, and then incubated with 50 *μ*g/ml propidium iodide (PI, Sigma-Aldrich) and 50 *μ*g/ml RNase A (Fermentas) for 30 min at room temperature in the dark. The stained nuclei were analyzed using a FACSCalibur flow cytometer with acquisition of 10,000 gated events. The DNA histograms were analyzed with the Flow software.

### 2.8. Transwell Invasion Assay

The frozen Matrigel at -20°C was dissolved at 4°C one day before the invasion experiment. On the second day, before gluing, 100 *μ*l PBS was added to the chamber, and it was left at room temperature for 30 min to fully soak the chamber. After the PBS was sucked out, it was dried naturally in the safety cabinet for about 20 min. 30 *μ*l diluted (1 : 5) glue was added into the chamber, and it was placed at 4°C for 1 h to balance. Then, the board with the chamber was incubated at 37°C for 4 h to allow the glue to solidify. Cells were digested with trypsin, centrifuged, and resuscitated in DMEM medium, cell count was performed, and cell concentration was adjusted to 4x10^5^/ml. Cell suspension of 0.1 ml was added to the compartment, and 0.6 ml was added to complete culture based on the lower well. The chamber was carefully placed into the orifice plate with medium with tweezers (avoid bubbles at the bottom), and it was placed in the incubator. The migration situation was observed every day, and the culture was generally stopped at 48 h. The compartment was removed, the supernatant was removed from the compartment, and the cells in the upper compartment was carefully wiped off with a wet cotton swab. At room temperature, the cells were slightly washed with PBS. 0.5 ml 4% paraformaldehyde was absorbed into a clean hole, it was put into a small chamber, and it was fixed at room temperature for 15 min. The invaded cells were the mean value of separate 6 fields, and the magnification times were of 100 folds.

RETRACTED

### 2.9. Vasculogenic Tube Formation Assay

Vasculogenic tube formation assays were performed as previously described [24]. Briefly, DU145 cells (3 × 104 cells), which are resuspended in 500 *μ*l of EBM-2 with 2% FBS, were seeded in 24-well cell culture plates (precoated with 100 *μ*l of Matrigel) and incubated for 22 h at 37°C. The tubes (closed areas surrounded by cells) were quantified with the Wimasis Image Analysis software by averaging the number of loops from four separate 20 × fields.

### 2.10. VEGF Secretion Assessment

VEGF release was assessed by a human-specific VEGF Quantikine ELISA Kit (R&D Systems, USA) according to the manufacturer's protocol.

### 2.11. *In Vivo* Tumorigenesis Assay

The treated DU145 cells (1 × 105 cells/3 *μ*l of DMEM) were injected into three groups of mice: (i) the DU145 group (no treatments, *N* = 20), (ii) the DU145-lenti-EGFP group (DU145 cells transfected with lenti-EGFP lentivirus, *N* = 58), and (iii) the DU145-lenti-EGFP-SNHG12-miR group (DU145 cells transfected with lenti-EGFP-SNHG12-miRLentivirus, *N* = 58). These cells were subcutaneously injected into the posterior flanks of 6-week-old male nude mice, and the tumor diameters were measured every three days. The tumor volume was calculated as the length × width^2^ × ½ mm^3^. The mice were sacrificed by CO_2_ inhalation to ameliorate animal suffering, and the tumors were collected and weighed. The protocol was approved by the Ethic Committee of the First Affiliated Hospital of Jinan University and the Sixth People's Hospital Affiliated with Shanghai Jiao Tong University, following the Committee Guidelines on the Use of Live Animals in Research and the National Institutes of Health Guide for the Care and Use of Laboratory Animals.

### 2.12. Statistical Analysis

Statistical analysis was performed using the SPSS 20.0 software (IBM SPSS, USA), and all experiments were performed at least three times to ensure the accuracy of the experiment. The tumor volumes are expressed as the mean ± standard error of the mean (SEM), and all the other values are expressed as the mean ± SD. Student's *t*-test or nonparametric Mann–Whitney *U* test was conducted to analyze the differences between the 2 groups, and multiple comparisons were assessed by one-way analysis of variance (ANOVA) followed by a Bonferroni post hoc test. A two-sided *P* value less than 0.05 indicated a statistically significant difference.

## 3. Results

### 3.1. SNHG12 Was Upregulated in PCa Tissues and Cell Lines

The expression level of SNHG12 were determined in PCa tissues and matched normal adjacent tissues from 85 patients (Table 1). We found that the expression of SNHG12 in PCa tissues was significantly higher than that in matched normal adjacent tissues (*P* < 0.05) (Figure 1(a)). The gene expression level of SNHG12 in several PCa cell lines (DU145, LNCAP, and PC-3) and normal human prostate stromal cell line (WPMY-1) was detected by qRT-PCR. We found that SNHG12 was significantly upregulated in the DU145 cell line compared with the normal human prostate stromal cell line (WPMY-1) and the other two human prostate carcinoma cell lines, LNCAP and PC-3 (Figure 1(b)). Therefore, we chose the DU145 carcinoma cell line as an *in vitro* model for functional study of SNHG12.

RETRACTED

### 3.2. Knockdown of SNHG12 Inhibited Proliferation of PCa Cells

Our results indicated that SNHG12 knockdown suppressed PCa cell proliferation and cell cycle progression. To investigate the function of SNHG12 in the proliferation of PCa cells, DU145 cells were transduced with lentiviral shRNA targeting the human SNHG12 gene (Figure 2(a)). Compared to the control group, the colony formation ability of DU145 cells was significantly decreased with SNHG12 knockdown (Figure 2(b)). The MTT assay showed that DU145 cell viability was also reduced by SNHG12 knockdown (Figure 2(c)). The cell cycle analysis of DU145 cells treated with knockdown of SNHG12 was performed by flow cytometry. Compared with the control group and the DU145+lenti-EGFP group, fewer DU145 cells transfected with lenti-EGFP-SNHG12-miR were in the G0/G1 phase, but more cells were in the S phase in the control group than in the SNHG12 knockdown group. The portion of DU145 cells in G2/M phase have no difference between the control group and the SNHG12 knockdown group (Figures 2(d) and 2(e)).

### 3.3. Knockdown of SNHG12 Promoted Early Apoptosis of PCa Cells

The function of SNHG12 in PCa cell apoptosis was analyzed by flow cytometry technique. Early apoptosis ration of DU145 cells in the SNHG12 knockdown group were significantly higher than that in control group, whereas the late apoptosis ratio of DU145 cells have no difference among the three groups. The results suggested that knockdown of SNHG12 significantly increased early apoptosis ratio of DU145 cells (Figures 3(a) and 3(b)).

### 3.4. SNHG12 Promoted PCa Cell Invasion

To further clarify the function of SNHG12 in the PCa cell invasion, we used a Transwell invasion assay. The Transwell invasion assay showed that the number of DU145 cells that migrated from the upper chamber to the lower chamber was markedly lower in the group stably transfected with lenti-EGFP-SNHG12-miR than in the untreated group or the group transduced with lenti-EGFP (*P* < 0.0001; Figures 4(a) and 4(b)).

RETRACTED

### 3.5. SNHG12 Might Have Affected Angiogenesis Tube Formation by PCa Cells

The effect of SNHG12 on vasculogenic tube formation was investigated. There were no significant differences in tube formation among the three groups (*P* > 0.05; Figures 5(a) and 5(b)). However, knockdown of SNHG12 significantly downregulated the expression of VEGF (Figure 5(c)). These results suggest that SNHG12 had no obvious effect on vasculogenic tube formation in prostate tumors but negatively affect secretion of VEGF.

### 3.6. SNHG12 Affected the Expression of Apoptosis-Related and Invasion-Related Proteins

The protein levels of the apoptosis-related molecules Bax, Bcl-2, cleaved caspase-3, and the cell invasion-related molecule MMP-9 were determined. Our western blot analysis indicated that the expression of cleaved caspase-3 was significantly upregulated in DU145 cells with SNHG12 knockdown (*P* < 0.05), although the expression of bcl-2 did not differ significantly among the three groups (*P* > 0.05; Figure 6(a)). In contrast, MMP-9 was markedly downregulated in the group of DU145 cells transfected with lenti-EGFP-SNHG12-miR compared with the other two groups (*P* < 0.05; Figure 6(b)). The PI3K/AKT signaling pathway plays a pivotal role in the invasiveness of PCa cells. Therefore, we also evaluated the effect of SNHG12 on AKT phosphorylation. Additionally, SNHG12 knockdown inhibited the expression of phosphorylated AKT (Figure 6(b)), although total AKT was not significantly different in the three groups (Figure 6(c)). The above-mentioned results suggested that SNHG12 knockdown suppressed the invasiveness of PCa cells via upregulating caspase-3 and downregulating MMP-9 and phosphorylated AKT.

### 3.7. SNHG12 Knockdown Inhibited Tumor Growth *In Vivo*

To further investigate the effect of SNHG12 on PCa *in vivo*, we established a nude mouse xenograft model with DU145 cells. DU145 cells were stably transfected with lenti-EGFP or lenti-EGFP-SNHG12-miR. Transfected cells or wild-type DU145 cells were subcutaneously inoculated into nude mice (*N* = 20 in DU145 group and *N* = 58 in DU145+lenti-EGFP or DU145+lenti-EGFP-SNHG12-miR groups). We found that body weights of nude mice were not significantly affected by the injection of DU145 cells (*P* > 0.05; Figure 7(a)). However, SNHG12 knockdown significantly inhibited tumor growth on the 28th day after inoculation (*P* < 0.05; Figure 7). Twenty-eight days after inoculation, the tumor weights and tumor sizes were significantly smaller in mice inoculated with DU145-lenti-EGFP-SNHG12-miR cells than in mice inoculated with wild-type DU145 cells or negative control DU145-lenti-EGFP cells (both *P* < 0.05; Figures 7(b)–7(d)). The results from the *in vivo* assay demonstrated that SNHG12 knockdown dramatically inhibited tumor growth.

RETRACTED

## 4. Discussion

Our study provides novel knowledge about the mechanism of how a lncRNA, SNHG12, is associated with PCa. Compared with previous similar studies [22, 23], we detected SNHG12 levels in tissues from PCa patients tissues and three PCa-derived-associated cells (LNCAP, DU145, and PC-3) as well as myofibroblast stromal cell line (WPMY-1 cells), by qRT-PCR. We revealed that there was a significant increase in SNHG12 expression in clinical PCa tissues and DU145 cells compared to matched normal adjacent tissues from patients and other cell lines investigated, which was in line with previous findings [23]. Upregulated SNHG12 expression has been reported in various other cancers, such as cervical cancer [21], hepatocellular carcinoma [24], and others [20]. Therefore, our findings support the idea that SNHG12 might be an oncogenic molecule in the development of these cancers, including PCa. SNHG12 can be a potential prognostic and diagnostic biomarker in PCa patients.

Our results of the MTT assay and colony formation assay showed that SNHG12 knockdown inhibited proliferation and cell cycle progression in PCa cells, in line with a recent study on PCa [22] and other cancer studies such as hepatocellular carcinoma [20, 24]. Uncontrolled cell proliferation and a dysfunctional cell cycle are key features during the tumorigenesis process of PCa [1], as of many other cancers [25]. It has also been confirmed that SNHG12 promotes the proliferation glioma cells by binding to HuR [26] and SNHG12 increases the expression of cell cycle-related proteins to accelerate cell growth in colorectal cancer [27]. In addition, the flow cytometry results showed that knockdown of SNHG12 expression significantly promoted early apoptosis in DU145 cells and upregulated the caspase-3, suggesting that knockdown of SNHG12 induced cell early apoptosis through the caspase signaling pathway, which is consistent with the functions of SNHG12 in NSCLC cells [28]. Previous studies have already reported that metastasis of cancer cells is the main cause of treatment failure in most patients with advanced cancer, and invasion is the first step that triggers cancer metastasis [29]. Herein, SNHG12 knockdown markedly suppressed PCa cell invasiveness and downregulated the expression of the cell invasion-related protein MMP-9, which suggested that SNHG12 promoted the DU145 invasion and probably participated in the metastasis of PCa. Additionally, angiogenesis is also a major factor that promotes tumor formation, as angiogenesis can provide better nutrition for tumor cells to promote their growth. Interestingly, we found that the knockdown of SNHG12 had no evident effect on vasculogenic tube formation in DU145 cells despite the fact that it could remarkably decrease secretion of VEGF, which is molecular playing a critical role in angiogenesis. The *in vivo* xenograft experiment demonstrated that SNHG12 knockdown inhibited prostate tumor growth. The above-mentioned results indicated that SNHG12 can be a potential therapy target in the treatment of PCa.

RETRACTED

Our results indicated that the AKT pathway was positively regulated by SNHG12, as found in studies of renal cell carcinoma [30]. Herein, downregulation of p-AKT expression was evident upon SNHG12 knockdown in DU145 cells. Similar downregulation of p-AKT after SNHG12 knockdown was also observed in studies of gastric cancers [31]. SNHG12 may promote PCa cell proliferation and cell cycle progression by activating the PI3K/AKT signaling pathway, the detailed mechanism requires further investigation.

In conclusion, our study demonstrated that SNGH12 was upregulated in PCa tissues and cells, and knockdown of SNGH12 inhibited the proliferation and invasion of PCa cells and suppressed the PCa growth which provided new evidence that SNHG12 could be a valuable biomarker for PCa diagnosis and prognosis and a potential target for PCa gene therapy. We encourage future studies to uncover more detailed mechanisms of the SNGH12 as a regulator of PCa and other cancers.

## Figures and Tables

**Figure 1:** Relative expression of SNHG12 in PCa tissues (a) and in different PCa cell lines (b) as detected by qRT-PCR. The data are reported as the means ± SD. The symbol “∗” indicates there is a significant difference between the pair of experiments (Student's *t*-test, *P* < 0.05).

**Figure 2:** Negative effects of SNHG12 knockdown on the proliferation of PCa cells, as shown by SNHG12 expression (a), colony formation abilities (b), MTT assays (c), cell cycle progression (d), and the associated statistical results (e) for three experiment groups: the control group (DU145 cells), empty vector group (DU145 cells transduced with lenti-EGFP), and SNHG12 knockdown group (DU145 cells transduced with lenti-EGFP-snhg12-miR). The data are reported as the mean ± SD. ∗∗*P* < 0.01, ∗∗∗*P* < 0.005, and ∗∗∗∗*P* < 0.0001 compared with the control group (Student's *t*-test).

**Figure 3:** Positive effects of SNHG12 knockdown on early apoptosis, as demonstrated by flow cytometric analysis (a), and the associated statistical results (b) for the three experiment groups: the control group (DU145 cells), empty vector group (DU145 cells transduced with lenti-EGFP), and SNHG12 knockdown group (DU145 cells transduced with lenti-EGFP-snhg12-miR). The data are reported as the means ± SD. The symbol “∗” indicates there is a significant difference between the pair of experiments (Student's *t*-test, *P* < 0.05).

RETRACTED

**Figure 4:** Significant negative effect ofSNHG12 knockdown on cell invasion, as determined by the Transwell invasion analysis (scale bar, 100 *μ*m) (a), and the associated statistical results (b) for the three experiment groups: the control group (DU145 cells), empty vector group (DU145 cells transduced with lenti-EGFP), and SNHG12 knockdown group (DU145 cells transduced with lenti-EGFP-snhg12-miR). ∗∗∗*P* < 0.0001 compared with the control group (Student's *t*-test).

**Figure 5:** Effects of SNHG12 knockdown on xxx, shown with images of vasculogenic tubes (scale bar, 100 *μ*m) (a), the number of branch points (b), and the concentrations of secreted VEGF (c) for the three experiment groups: the control group (DU145 cells), empty vector group (DU145 cells transduced with lenti-EGFP), and SNHG12 knockdown group (DU145 cells transduced with lenti-EGFP-snhg12-miR). The symbol “∗” indicates there is a significant difference between the pair of experiments (Student's *t*-test, *P* < 0.05).

**Figure 6:** The protein expression of apoptosis-related protein (Bax, Bcl-2, caspase-3, p-Akt, and total AKT) and invasion-related protein MMP-9 In PCa cell transfected with lenti-EGFP-SNHG12-miR. (a) The protein expression of Bcl-2, Bax, and caspase-3, (b) the protein expression of MMP-9, p-AKT, and AKT, and (c) relative protein level of Bax. Bcl-2, caspase-3, MMP-9, p-AKT, and AKT in the three experiment groups: the control group (DU145 cells), empty vector group (DU145 cells transfected with lenti-EGFP), and SNHG12 knockdown group (DU145 cells transfected with lenti-EGFP-SNHG12-miR).

**Figure 7:** Significant negative effect ofSNHG12 knockdown on PCa tumor progression in nude mice, as shown with body weights (a), tumor weights (b), tumor volumes (c), and tumor images (d) for mice in the three groups: the control group (injected with DU145 cells), empty vector group (injected with DU145 cells transduced with lenti-EGFP), and SNHG12 knockdown group (injected with DU145 cells transduced with lenti-EGFP-snhg12-miR). The data are reported as the mean ± SD. ∗∗*P* < 0.01 compared with the control group (Student's *t*-test).

**Table 1:** The clinicopathological information of recruited cases.

Variable	Total no. (%)
No. of cases	85
Median age (y, range)	66 (47-85)
Median PSA (ng/ml, range)	7.84 (1.80-10.00)
Median FPSA (ng/ml, range)	0.87 (0.12-1.89)
Biopsy Gleason sum, *n*	
≤6	85 (100%)
AJCC-T stage, *n*	
T1c	0 (0%)
T2a	36 (42.35%)
T2b	24 (28.24%)
T2c	25 (29.41%)
T3	0 (0%)
Pathological Gleason sum, *n*	
≤6	62 (72.94%)
3 + 4	12 (14.12%)
4 + 3	11 (12.94%)
≥8	0 (0%)
Surgical margin, *n*	
Negative	80 (94.12%)
Positive	5 (5.88%)
Lymph node invasion, *n*	
Negative	83 (97.65%)
Positive	2 (2.35%)
Biochemical recurrence, *n*	7 (8.24%)
Clinical progression, *n*	2 (2.35%)
Follow-up months, median (range)	48 (8-96)

RETRACTED

## Data Availability

All data, models, and code generated or used during the study appear in the submitted article.
